# Melanoma Molecular Subtypes and Development of Prognostic and Immunotherapy-Related Genetic Characteristics by Ferroptosis Gene Analysis

**DOI:** 10.1155/2022/2992939

**Published:** 2022-04-26

**Authors:** Libin Xu, Yu Zhang, Ting Liu, Luqiang Wang, Zhenguo Zhao, Xinxin Zhang, Xiaoyang Li, Wence Wu, Shengji Yu

**Affiliations:** ^1^Department of Orthopedic Surgery, National Cancer Center/National Clinical Research Center for Cancer/Cancer Hospital, Chinese Academy of Medical Sciences and Peking Union Medical College, 17 Panjiayuan Nanli, Chaoyang District, Beijing 100021, China; ^2^Department of Immunology, National Cancer Center/National Clinical Research Center for Cancer/Cancer Hospital, Chinese Academy of Medical Sciences and Peking Union Medical College, Beijing 100021, China

## Abstract

The dissimilarity is a major problem in clinical therapy of skin cutaneous melanoma (SKCM). Objective and reproducible classification systems may help decode SKCM heterogeneity. ConsensusClusterPlus was used to establish a stable immune molecular classification based on ferroptosis-related genes that had been acquired from FerrDb. Moreover, the prognosis, somatic mutations, immune microenvironment characteristics, functional enrichment, and clinical responsiveness to the immune checkpoint blockade of different subtypes in two independent melanin datasets were compared. Kaplan-Meier curves, univariate, multivariate, least absolute contraction, and selection operator (LASSO) Cox regression analysis were used to develop a molecular model for predicting survival, which was verified by a nomogram on the basis of independent prognostic indicators. Two molecular subtypes (C1 and C2) for SKCM were first identified according to ferroptosis-related genes; C1 showed a poor prognosis, with lower infiltration degree of immune cells and TIED score and higher homologous recombination defects, fraction altered, the number of segments, and copy number amplification and deletion. These characteristics of C2 were the opposite of C1. A ferroptosis-related prognosis risk score (FPRS) model was constructed using 6 of 463 genes with differential expression between C1 and C2. This model splits patients into low- and high-risk cohorts. There were significant differences in the infiltration and proportion of immune cells, immune checkpoint gene expression, responsiveness to immune checkpoint therapy, and sensitivity to chemotherapeutic medications between low- and high-risk cohorts. This model was an independent prognostic marker for SKCM and has a high AUC. In summary, we have identified two subtypes of SKCM with different molecular and immune characteristics on the basis of ferroptosis-related genes and further developed and verified an FPRS model, which might independently serve as a prognostic marker for SKCM.

## 1. Introduction

Skin cutaneous melanoma (SKCM) has been identified as a skin cancer whose origin is the malignant transformation of melanocytes. Superficial diffusion, nodular, and malignant freckles are the three main histological types of SKCM [1]. By 2020, 4.2% of the global population suffered from SKCM [2]. SKCM accounts for about 5% of all skin cancers but more than 2/3 of all skin cancer-related mortality. Patients with topical or regional lesions exhibited five-year survival rates of 98 percent and 64 percent, respectively, but those experiencing metastatic melanoma exhibited extremely unfavorable survival rates of 23 percent [3].

Recent breakthroughs in scientific knowledge of the molecular and cellular processes behind carcinogenesis, metastasis, and immune evasion have resulted in the advent of novel therapeutic approaches, such as targeted treatment and immunotherapy [4]. However, responses to these treatments still vary among patients. To optimize current targeting and immunotherapy modalities, it is necessary to identify novel therapeutic targets and approaches for the accurate categorization of melanoma patients [5].

Ferroptosis is known as the process in which regulatory cells die as a result of iron buildup and lipid peroxidation [6]. Ferroptosis also exhibits distinct bioenergy and morphological features, such as mitochondrial atrophy, increased density of the mitochondria membrane, membrane integrity damage, and intracellular NADH depletion, but does not include ATP levels [7]. Ferroptosis has been found to participate in the pathogenesis of a variety of clinical disorders, such as neurodegeneration, ischemic tissue injury, and infection [8]. Ferroptosis is also associated with many types of cancer. TP53 induces iron death resistance in colorectal cancer via the inhibition of the dipeptidyl peptidase 4 (DPP4) activity in a manner that is transcription-independent [9]. FSP1 in lung cancer has been recognized as a crucial constituent of the nonmitochondrial CoQ antioxidant system, which endows cells with ferroptosis resistance in parallel with glutathione-based GPX4 pathway [10]. Recent studies showed the great potential of ferroptosis reagent in cancer treatment, especially in overcoming chemotherapy resistance during cancer treatment [7]. It is reported that iron death inducer erastin could enhance the responsiveness of acute myeloid leukemia cells to chemotherapeutic drugs cytarabine and ara-C and doxorubicin and adriamycin [11] and increase the sensitivity of cancer cells to adriamycin and actinomycin D in rhabdomyosarcoma [12]. Therefore, the study of ferroptosis in malignant tumors is of great significance for cancer treatment.

At present, there are several system biology methods to identify biomarkers related to skcm prognosis and construct gene features. Niu et al. [13] identified a 4-gene signature in pyrosis-related gene expression profile by LASSO regression analysis, and Fei and Chen [14] identified a 4-gene signature in autophagy-related gene expression profile by Cox regression analysis. All two groups of authors tested their gene signature in internal and external data sets but did not verify the clinical data, which means that identifying robust gene signature is still a challenge. Based on the above background, the present research is aimed at investigating the molecular subtypes of SKCM in Gene Expression Omnibus (GEO) and The Cancer Genome Atlas (TCGA) according to ferroptosis-related genes and at developing a ferroptosis-related prognosis risk score (FPRS) model, to examine the prognostic significance of this model in patients with SKCM.

## 2. Materials and Methods

### 2.1. Research Population and Data Processing

Complete public data of metastatic melanoma were downloaded from TCGA and GEO (GSE69504 [15], GSE54467 [16], and GSE22153 [17]). Specifically, TCGA-SKCM contained 358 metastatic samples, and GSE69504, GSE54467, and GSE22153 had 188, 79, and 54 metastatic SKCM samples, respectively. In addition, data for SKCM immunotherapy came from GSE78220 [18] and GSE91061 [19] data sets. Ferroptosis marker genes were searched in the public database FerrDb [20], and a sum of 11 genes was integrated for follow-up assessment. Supplementary figure 1 shows the workflow of this study.

### 2.2. Consensus Clustering of Genes Involved in Ferroptosis

ConsensusClusterPlus [21] was used to construct a consistency matrix on the basis of the expression profile of ferroptosis-related genes. 500 bootstraps were conducted utilizing the PAM algorithm, with “canberra” as the measurement distance, and each bootstrap procedure comprised 80 percent of the patients from the training set. The consistency matrix, as well as the consistency cumulative distribution function, was calculated for the purpose of determining the ideal number of clusters.

### 2.3. Creation and Verification of Ferroptosis-Related Prognosis Risk Score (FPRS) Model

For the purpose of establishing a predictive risk signature model that is based on genes associated with ferroptosis, a univariate Cox regression analysis was carried out, utilizing the coxph function to filter DEGs across subtypes. Then, the DEGs between subtypes were filtered by LASSO regression analysis and Akaike information criterion (AIC) for the second and third times, respectively. The coefficient (*β*) calculated by multiple Cox regression was used to characterize the weight to construct an FPRS model. With the aid of the median risk scores, the samples in the training and verification sets were classified into distinct groups. The Kaplan-Meier curve was utilized to probe into the survival rates of various groups, and the significance of the differences was assessed utilizing the logarithmic rank test. Time-dependent receptor operating characteristic (ROC) curves were plotted to calculate AUC. FPRS was also subjected to a multivariate Cox regression analysis according to the risk score and clinical characteristics to determine if it independently served as a prognostic predictor of SKCM.

### 2.4. Functional Enrichment Analysis

To interpret differences in enrichment pathways among different molecular subtypes, all candidate gene sets in the Hallmark database [22] were employed in the gene set enrichment analysis (GSEA) [23] and shown by enrichplot. DEGs between different molecular subtypes were screened by Limma (threshold: multiple variations > 2 and *p* < 0 01), and then, Gene Ontology (GO) and Kyoto Encyclopedia of Genes and Genomes (KEGG) pathway enrichment analyses on the DEGs were carried out utilizing “clusterProfiler” [24] R software.

### 2.5. Analysis of Immune Characteristics

CIBERSORT algorithm was first introduced, as it can distinguish 22 leukocyte subgroups, such as myeloid subsets, NK cells, plasma cells, naïve and memory B cells, and 7 T cell types [25]. CIBERSORT was applied to study the distribution and invasion of 22 different immune cells in SKCM tissues. At the same time, the immune characteristics of each molecular subtype were also evaluated by the ESTIMATE [26] software in “Stromal Score,” “Immune Score,” and “ESTIMATE Score.”

### 2.6. Construction of Nomogram

Independent predictors were identified utilizing multivariate Cox regression. To assess the risk assessment and survival probability of SKCM patients, the alignment and calibration maps were established through combining FPRS and other clinicopathological features using the “rms” R software. Decision curve analysis (DCA) was performed for the purpose of comparing the clinical utility of the nomogram with that of FPRS.

### 2.7. Statistical Analysis

The “survminer” module of the R package was used for performing univariate and multivariate Cox regression analyses. The ROC curve was generated by “timeROC.” The forest plot created utilizing the R software was drawn to visually display clinical variables and risk score and survival findings of multivariate Cox analysis. Unless otherwise specified, the *p* value on both sides or adjusted *p* value < 0.05 was taken as the threshold signifying statistical significance.

## 3. Results

### 3.1. Consensus Clustering Based on Ferroptosis-Related Gene Identified Two Subtypes of SKCM

After conducting a univariate Cox analysis of 111 genes associated with ferroptosis, 31 genes were observed to be significantly correlated with the prognosis of SKCM. Based on these 31 genes, 358 SKCM samples were clustered by ConsensusClusterPlus. According to the CDF Delta area, *k* = 2 had the highest clustering stability. Therefore, SKCM samples were divided into two molecular subtypes (Figures 1(a)–1(c)). Classification information of each sample in TCGA dataset is shown in Supplementary Table 1. Different overall survival (OS) of the two subtypes was observed that the OS of Cluster 1 (C1) was substantially shortened in contrast with that of Cluster 2 (C2), meaning that C1 was more dangerous (Figure 1(d)). In TCGA, substantial differences were observed between the 2 distinct molecular subtypes in the patients' survival status, and the death rate of patients with a poor prognosis of the C1 subtype was remarkably elevated as opposed to that of the C2 subtype having a good prognosis (Figure 1(e)). The same was found in GSE65904 (Figures 1(f) and 1(g)).

### 3.2. Differences in Molecular Characteristics and Energy Function between Two Types of SKCM Subtypes

To distinguish the molecular characteristics between the two SKCM subtypes, aneuploidy score, homologous recombination defects, altered fractions, tumor mutation burden, and proportion of segments of different subtypes were analyzed. According to the result of the Wilcoxon test, C1 showed homologous recombination defects, fraction altered, and number of segments higher than C2, with a significant difference (Figure 2(a)). Then, the correlations between gene mutation and copy number variation and two subtypes were analyzed, and we found a significant correlation between subtype and gene mutation. BRAF was highly mutated in both subtypes, but it was mutated more frequently in C2 (up to 59%). The mutation frequency of MUC5B (27% vs. 14%) and ENPEP (26% vs. 11%) in the C1 subgroup was substantially elevated in contrast with that in the C2 subgroup. Copy number variation (copy number amplification and copy number deletion) in C1 was also elevated as opposed to that in C2 (Figure 2(b)). GSEA analysis was performed to confirm whether there were differentially regulated pathways in different isoforms.  Figure 3(a) shows the Hofmann pathway normalized enrichment score (NES) heat maps calculated by comparing C1 and C2 (error detection rate (FDR) < 0.05). With regard to the TCGA-SKCM cohort, 20 pathways in the C2 subclass were activated, and 1 pathway was inhibited. In the GSE65904 cohort, C2-activated pathways were implicated in various pathological characteristics and behaviors of cancer, including immunity (interferon-gamma response, allograft rejection, inflammatory response, and complement), metastasis (epithelial-mesenchymal transition), and proliferation (apoptosis, MYC target, G2M checkpoint, and mitotic spindle) (Figures 3(b) and 3(c)).

### 3.3. Immune Microenvironment Characteristics of Different Molecular Subgroups

To clarify the differences in immune microenvironment between two subpopulations, the GSE65904 and TCGA-SKCM cohorts were analyzed utilizing the CIBERSORT algorithm to determine the degree of immune infiltration. Among the 12 immune cells in the TCGA-SKCM cohort showing significant differences between the two subtypes, the proportion of eosinophils, naive B cells, M0 and M2 macrophages, helper follicular T cells, and resting NK cells in C1 was considerably elevated in contrast with that in C2, while the predicted levels of memory T cell, gamma delta T cells, regulatory T cells, activated memory CD4 T cells, CD8 T cell, and M1 macrophages in C2 were substantially elevated as opposed to that in C1 (Figure 4(a)). Three kinds of tumor environment scores evaluated by ESTIMATE in C2 were considerably elevated in contrast with those in C1 (Figure 4(b)). In the GSE65904 cohort, 6 of 22 kinds of immune cells showed a statistical difference between C1 and C2. The proportion of plasma cells, helper T cells, M0 macrophages, and eosinophils in C1 was noticeably higher than that in C2. The proportion of resting memory CD4 T cells and memory B cells was substantially elevated in C2 (Figure 4(c)). In line with the findings of the TCGA-SKCM cohort, ESTIMATE, immune, and stromal scores in C2 were considerably higher in contrast with the scores in C1 (Figure 4(d)). These findings illustrated that the degree of immune infiltration of C2 was higher.

### 3.4. Prediction of SKCM Molecular Subgroup Response to Immune/Chemotherapy

The different patterns of immune infiltration in different classes of SKCM subgroups required further study of patient response to immunotherapy. Therefore, we obtained immune checkpoint data from HisgAtlas database [27] and analyzed the differences in the expression in immune checkpoint genes between the 2 subtypes in two independent cohorts. Figures 5(a) and 5(b) illustrate that the immune checkpoint gene with a large bottom plate number was highly expressed in subtype C2. The TIDE (http://tide.dfci.harvard.edu/) software was utilized to evaluate the potential clinical effects of immunotherapy on different melanoma subgroups. Among the TCGA and GSE65904 cohorts, C2 had the highest predicted TIDE score, suggesting that this subtype had a greater likelihood of immune evasion and was less likely to benefit from immunotherapy (Figures 5(c) and 5(d)). On the other hand, the responses of C1 and C2 to chemotherapeutic drugs paclitaxel, cisplatin, vinblastine, and temozolomide were analyzed, and it was observed that C2 was more sensitive to paclitaxel and temozolomide, while patients in the C1 subtype were more sensitive to cisplatin (Figure 5(e)).

### 3.5. Functional Enrichment Analysis and FPRS Model Identification Based on the DEGs between C1 and C2

Through the analysis of gene differences between C1 and C2, a sum of 464 DEGs was obtained, of which 415 DEGs were downmodulated and 49 that upmodulated. From GO analysis, we observed the DEGs between C1 and C2 were enriched in cancer immunity-related GO terms, such as regulation of leukocyte activation, T cell activation, modulation of the adhesion of leukocyte cell−cell, migration of leukocytes, activation of lymphocytes, modulation of the activation of T cells, MHC protein complex, and the activities of cytokines and cytokine receptors, as well as the binding of chemokine receptors (Figure 6(a)). The findings from KEGG analysis also demonstrated that DEGs were linked to immune regulation pathway, including cell adhesion molecules, phagosome, Th1, Th2, and Th17 cell differentiation, and hematopoietic cell lineage (Figure 6(b)). 353 (32 were “risk” genes and 321 were “protective” genes) out of the 463 DEGs had significant effects on the prognosis of SKCM (Figure 6(c)). After conducting LASSO COX analysis and AIC-based filtering, an FPRS model composed of TFAP2C, LIF, IFITM1, GBP4, PAEP, and KIT was established (Figures 6(d)–6(f)). From MsigDB database [22], the ferroptosis pathway was obtained from Hallmark gene sets. The enrichment score of ferroptosis pathway of each sample was calculated by ssGSEA method. The correlation between the expression of six genes and the enrichment score of ferroptosis pathway was further calculated. It was observed that GBP4, IFITM1, TFAP2C, and LIF were significantly positively correlated with ferroptosis pathway (Supplementary Figure 2A). In addition, we also analyzed the expression differences of these six genes in C1 and C2 subtypes. It can be observed that GBP4, IFITM1, TFAP2C, and LIF are significantly overexpressed in C2, and KIT and PAEP are significantly overexpressed in C1 (Supplementary Figure 2B).

### 3.6. Verification of FPRS Model

According to the samples in the FPRS model, the samples in TCGA-SKCM were classified into low- and high-risk groups. The patient's survival status distribution demonstrated that the increase of FPRS was inversely associated with the survival time of patients and had a positive association with the number of death cases. The low expression levels of TFAP2C, LIF, IFITM1, and GBP4 were associated with a high risk, which could serve as protective factors, while a high expression of PAEP and KIT genes was associated with elevated risk and was therefore considered to be risk factors (Figure 7(a)). The results of the Kaplan-Meier survival curve illustrated that death risk was substantially elevated in the high-risk SKCM samples in contrast with those with a low-risk (Figure 7(b)). Time-dependent ROC curves were utilized to calculate the area under the curve (AUC) at different time points, and AUC was 0.67, 0.71, and 0.75 for one-, three-, and five-year survival, indicating that the FPRS model had a good predictive value in long-term follow-up of SKCM (Figure 7(c)). In the three externally validated cohorts, patients having high-risk scores exhibited a significantly greater chance of premature decrease in contrast with those having low-risk scores (Figures 7(d), 7(f), and 7(h)). In the GSE65904 cohort, the AUC in the time-dependent ROC at one, three, and five years reached 0.7, 0.72, and 0.65, respectively (Figure 7(e)). In the GSE54467 cohort, the ferroptosis risk score had AUC values of 0.72, 0.63, and 0.67 for one, three, and five years (Figure 7(g)). For the GSE22153 cohort, the AUCs for OS were 0.66, 0.7, and 0.78 for one, three, and five years, suggesting an increased predictive capability in long-term follow-up (Figure 7(i)).

### 3.7. Variation in Immune Infiltration and Immunotherapy Responses across Low- and High-FPRS Samples

The proportion of 22 distinct immune cells in SKCM was anticipated for the purpose of distinguishing differences in immune infiltration between low- and high-risk groups. The contents of M0 and M2 macrophages and CD8 T cells were the highest in 22 immune cells (Figure 8(a)). The landscape of 22 different immune cells between low- and high-risk groups is in Figure 8(b). Specifically, 10 out of 22 immune cells showed substantial differences in the infiltration ratio between high- and low-risk samples. The high-risk group contained more eosinophils, M2 macrophages, resting NK cells, resting memory CD4 T cells, resting mast cells, and naive B cells, and the levels of M1 macrophages, active memory CD4 T cells, and CD 8 T cells in low-risk samples were considerably elevated as opposed to that in high-risk samples (Figure 8(c)). The differences of immune cell components in low- and high-risk samples were reflected in the heat map (Figure 8(d)). According to the calculation results of Pearson correlation analysis, 10 out of 22 immune cells were significantly correlated with FPRS, which were exactly the 10 kinds of immune cells with substantial differences in infiltration in low- and high-risk groups shown in Figure 8(b) (Figure 8(e)).

To some extent, the immune microenvironment could reflect the response to immunotherapy, thereby the correlation between FPRS and common immune checkpoints PDCD1, CTLA4, and CD274 (PD-L1) was further analyzed. The findings demonstrated that FPRS was substantially negatively correlated with all the three immune checkpoints; that is, a higher FPRS was negatively related to the expression of CTLA4, PD-L1, and PDCD1 and indicated a less active clinical response to immunosuppressant therapy (Figures 9(a)–9(c)). Then, melanoma anti-PD-1 (GSE78220) data were included, and the sample scores were calculated according to the FPRS model. The findings illustrated considerable differences in FPRS scores between different clinical responsiveness statuses of anti-PD-1 therapy, in which the FPRS scores of patients with response to immunotherapy were significantly lower than those with response status of PD, indicating that a higher FPRS score was associated with a less active response to anti-PD-1 immunotherapy (Figure 9(d)). Similarly, FPRS model calculation and grouping of melanoma samples in GSE78220 showed a shortened survival duration among the high-risk group in contrast with the low-risk group (Figure 9(e)). The AUC in the ROC was found to be 0.68, 0.81, and 0.85, for at 0.5, 1, and 2 years, respectively (Figure 9(f)).

### 3.8. Development of Nomogram Model for FPRS Combined with Clinicopathological Features

To evaluate the independence of HPRS, multivariate and univariate Cox regression analyses were performed, and FPRS was verified as the most remarkable independent prognostic marker (Figures 10(a) and 10(b)). The nomogram established by combining FPRS with other clinicopathological features showed that FPRS had the greatest contribution to the prediction of survival rate (Figure 10(c)). The calibration curves showed that the predicted curves at the calibration point 1, 3, and 5 years were nearly the same as the standard curves, suggesting that the nomogram can effectively predict the OS of SKCM (Figure 10(d)). According to DCA, the nomogram showed comparable clinical applicability similar to FPRS (Figure 10(e)), and it had the highest AUC value (Figure 10(f)).

## 4. Discussion

Metastatic melanoma shows significant heterogeneity, including the rate of disease progression and location of metastatic lesions. 1/3 of patients with metastatic melanoma at their first diagnosis have a multifocal and rapidly progressive disease and are whether through targeted therapy or immunotherapy, but it is largely unable to achieve long-term remission [28]. Thereby, new therapeutic strategies should be developed to attack tumor cells by exploiting the weaknesses of such tumors [29].

In fact, considerable efforts have been made in the design and development of ferroptosis-induced anticancer drugs [30]. At present, the majority of research reports on ferroptosis emphasize the identification of iron death inducers, such as small molecules, nanomaterials, and genes that can be used as cancer treatment strategies [31]. Here, we studied SKCM through ferroptosis-related genes. In view of the heterogeneity of melanoma, we first clustered the SKCM in TCGA according to ferroptosis-related genes and successfully divided SKCM into two subtypes. Subtype C1 was characterized by poor prognosis, high variation of homologous recombination defects, altered fraction, number of segments, gene creep frequency and copy number, and relatively low degree of immune infiltration in the tumor microenvironment, which will facilitate tumor growth [6]. Compared with C1, C2 had a significant survival advantage, as it showed a higher degree of overall immune infiltration in the tumor microenvironment and was less likely to benefit from immunotherapy but was sensitive to paclitaxel and temozolomide.

Based on the DEGs between different subtypes, we developed an FPRS model composed of TFAP2C, LIF, IFITM1, GBP4, PAEP, and KIT. TFAP2C is a well-recognized affiliate belonging to the AP-2 transcription factor family. The relationship between TFAP2C and the progression of SKCM has been previously found in Elisa Penna's reports, and its expression was inhibited by miR-214 [32]. TFAP2C is also an important prognostic medium for SKCM through regulating the expression of ECM1 [33] and has been considered as a protective factor for SKCM in our study. According to the findings of Maruta et al., LIF might be a viable and effective drug target for bone metastasis therapy in SKCM [34]. Studies also analyzed the mechanism of LIF in SKCM. Specifically, LIF and p21 act on the downstream of TGF *β* in SKCM to regulate cell cycle arrest and cell death [35]. In tumor tissues, LIF has been shown to be overexpressed and is demonstrated to independently serve as a predictive indicator for patients with various malignant tumors, such as gastric cancer, colorectal cancer, esophageal adenocarcinoma, and gallbladder carcinoma [36]. According to the current consensus, GBP expression is primarily stimulated by IFN*γ* in many kinds of cells and has been identified as significantly positively correlated with infiltrating immune cells of SKCM [37]. PAEP protein secreted by SKCM cells could suppress the cytotoxicity, proliferation, and activation, of T lymphocytes, which may partly elucidate the process of immunological tolerance caused by melanoma cells in tumor microenvironment [38]. KIT has been discovered as a potential therapeutic target in the treatment of metastatic melanoma [39].

The FPRS model can divide SKCM samples into low- and high-risk groups with different survival outcomes. In case when comparing the low-risk group to the high-risk group, it was found that there were significant differences in the infiltration and proportion of immune cells, the immune checkpoint gene expression, responsiveness to immune checkpoint therapeutic interventions, and responsiveness to chemotherapy agents. The FPRS model might thus have a possible function in anticipating the clinical response of SKCM to immunotherapeutic treatment. In addition, the FPRS model was also found to independently serve as a prognostic marker for SKCM.

To conclude, on the basis of genes correlated with ferroptosis, two types of SKCM molecular subtypes with different molecular and immune characteristics were established, and a reliable FPRS model was developed as an independent factor for SKCM survival prediction. Furthermore, the FPRS model also showed a potential association between ferroptosis and SKCM immune characteristics and immunotherapy responses. These findings could deliver crucial implications for the development of new therapeutic options for SKCM.

## Figures and Tables

**Figure 1:** SKCM subtypes were identified by consensus clustering. (a) CDF curves of SKCM samples in TCGA cohort. (b) CDF delta area curves of SKCM samples in TCGA cohort. Delta area curve of the consensus clustering, demonstrating the degree of variance in the area under the cumulative distribution function (CDF) curve for every classification number *k* in contrast with *k* − 1. The horizontal axis denotes the classification number *k*, while the vertical axis denotes the difference in the area under the CDF curve compared to the horizontal axis. (c) The consensus matrices of the TCGA for *k* = 2. (d) The Kaplan-Meier curves of patients with two subtypes of TCGA-SKCM. (e) Analysis of the difference of survival ratio between the two subtypes in TCGA-SKCM. (f) OS analysis between C1 and C2 in GSE65904. (g) The proportion of death and survival status between C1 and C2 in GSE65904 was analyzed. The bottom part represents the percentage, whereas the top part represents the statistical significance of the distribution difference between the two groups.

**Figure 2:** Analysis of molecular characteristics and functional differences between C1 and C2. (a) Wilcoxon test was used to analyze differences of aneuploidy score, homologous recombination defects, altered fraction, number of segments, and tumor mutation burden between C1 and C2 subgroups. (b) Copy number variation and somatic mutation of different subclasses in the TCGA-SKCM cohort were analyzed by the Fisher test. ^∗^*p* < 0.05; ^∗∗^*p* < 0.01; ^∗∗∗^*p* < 0.001; ^∗∗∗∗^*p* < 0.0001.

**Figure 3:** Differences biological pathway between two types of SKCM subtypes. (a) Heat map displaying the normalized enrichment scores (NESs) of Hallmark pathways, which were obtained by comparing C1 with C2. (b) The top 10 pathways enriched by C2 compared to C1 in the TCGA cohort. (c) Compared with C1, activated and inhibited top 10 pathways in C2 in the GSE65904 cohort.

**Figure 4:** Immune characteristics analysis of C1 and C2 in different cohorts. (a) The differences in the infiltration of 22 distinct immune cells between C1 and C2 in the TCGA-SKCM cohort. (b) In the TCGA-SKCM, differences between C1 and C2 in the three tumor microenvironment scores were assessed by ESTIMATE in the TCGA-SKCM cohort. (c) The differences in the infiltration of 22 distinct immune cells between C1 and C2 in the GSE65904 cohort. (d) The differences in ESTIMATE, immune, and stromal scores between C1 and C2 in the GSE65904 cohort.

**Figure 5:** Prediction of immuno/chemotherapeutic response. (a) Immune checkpoint molecules of C1 and C2 expressed differently in the TCGA-SKCM cohort. (b) The difference in the immune checkpoint molecule expression between two subtypes in the GSE65904 cohort. (c) TIDE score differences between C1 and C2 and the difference of immunotherapy predicted efficacy in the TCGA-SKCM cohort. (d) Difference of TIDE score and *t* immunotherapy predicted efficacy between the two subtypes in the GSE65904 cohort. (e) The box plots demonstrated the estimated IC50 for cisplatin, vinblastine, paclitaxel, and temozolomide in TCGA-SKCM.

**Figure 6:** Functional enrichment analysis of DEGs and characterization of the FPRS model between the two subgroups. (a) Enrichment findings of GO molecular function (MF), GO cellular component (CC), and GO biological process (BP) of DEGs between subtypes in TCGA cohort. (b) In the TCGA cohort, KEGG analysis of DEGs between C1 and C2. (c) A total of 353 promising candidates were identified among the DEGs. (d) The LASSO coefficient spectrum of genes that significantly affected the prognosis of SKCM. (e) Selection of 5-fold cross-validation parameters in LASSO model. (f) LASSO Cox coefficient distribution of 6 ferroptosis-related genes in the FPRS model.

**Figure 7:** Verification of the prognostic capability of the FPRS model in the training and external validation sets. (a) FPRS arrangement, expression of 6 genes, and survival status in the FPRS model of samples in TCGA-SKCM cohort. (b) Kaplan-Meier survival curve of low- and high-risk samples in TCGA-SKCM cohort. (c) Time-dependent ROC curves were utilized to calculate AUC at different time points. (d) The Kaplan-Meier survival curve of the SKCM sample in the GSE65904 cohort. (e) In the GSE65904 cohort, the AUC in the time-dependent ROC at one, three, and five years. (f) Kaplan-Meier survival curves of SKCM samples in the GSE54467 cohort. (g) The AUC of the FPRS in the GSE54467 cohort for 1, 3, and 5 years. (h) Kaplan-Meier analysis of GSE22153 SKCM patients. (i) ROC curves showed the predictive capability of the FPRS model.

**Figure 8:** Association of FPRS with immune cell infiltration. (a) Proportion of 22 different immune cells in samples from the TCGA-SKCM cohort. (b) Bar plot showed the levels of immune cell infiltration in the low- and high-FPRS groups. (c) The predicted proportion difference of 22 different immune cells between high- and low-FPRS samples. (d) Heat map illustrated immune cell distributions in low- and high-FPRS samples. (e) In the TCGA-SKCM cohort, a Pearson correlation analysis was performed between FPRS and immune cells. ^∗^*p* < 0.05; ^∗∗^*p* < 0.01; ^∗∗∗^*p* < 0.001.

**Figure 9:** Prediction immunotherapeutic response between low- and high-FPRS groups. (a) Correlation between FPRS and PDCD1 in TCGA-SKCM cohort. (b) Correlation between FPRS and immune checkpoint gene CTLA4 in TCGA-SKCM cohort. (c) Correlation between FPRS and PD-L1 expression in TCGA-SKCM cohort. (d) Differences in FPRS for different clinical responsiveness states to anti-PD-1 therapy in the GSE78220 cohort, where PD represents a progressive disease, PR represents a partial response, and CR represents a complete response. (e) In GSE78220, the OS of the low- and high-FPRS groups. (f) The AUC in the ROC at 0.5, 1, and 2 years.

**Figure 10:** A nomogram for anticipating the prognosis of samples according to HPRS and clinical characteristics. (a, b) The independent prognostic variables for SKCM were determined utilizing multivariate and univariate Cox regression analyses. (c) To estimate the survival rates of SKCM samples, a nomogram was constructed utilizing HPRS and clinical characteristics. (d) Calibration diagrams for anticipating SKCM OS at 1, 3, and 5 years. (e) DCA of OS-related nomogram in SKCM. (f) Nomogram, FPRS, and clinical variables predicted AUC for OS.

## Data Availability

The data used to support the findings of this study are included within the article.

## Supplementary Materials

Supplementary Materials Supplementary Figure 1: workflow. Supplementary Figure 2: expression relationship of six key genes: (A) correlation between six key genes and iron death pathway; (B) the expression and distribution of six key genes were different from those in C1 and C2 subgroups. Supplementary Table 1: classification information of each sample in TCGA dataset.
